# Upregulation of OIP5-AS1 Predicts Poor Prognosis and Contributes to Thyroid Cancer Cell Proliferation and Migration

This article has been retracted.

**DOI:** 10.1016/j.omtn.2019.11.036

**Published:** 2020-01-11

**Authors:** Qiuli Li, Weichao Chen, Rongzhen Luo, Zhiyi Zhang, Ming Song, Wenkuan Chen, Zhongyuan Yang, Yuanzhong Yang, Zhuming Guo, Ankui Yang

**Affiliations:** 1 Department of Head and Neck Surgery, Sun Yat-sen University Cancer Center, State Key Laboratory of Oncology in South China, Collaborative Innovation Center for Cancer Medicine, Guangzhou 510060, China; 2 Department of Pathology, Sun Yat-sen University Cancer Center, State Key Laboratory of Oncology in South China, Collaborative Innovation Center for Cancer Medicine, Guangzhou 510060, China

**Keywords:** OIP5-AS1, Wnt/β-catenin signaling, proliferation, migration, thyroid cancer

## Abstract

As a common malignancy, thyroid cancer mainly occurs in the endocrine system. There have been accumulating studies on therapeutic methods of thyroid cancer, but its internal molecular mechanism is still not fully understood. Long noncoding RNA (lncRNA) OIP5-AS1 was confirmed as an oncogene and related to poor prognosis in various cancers. Nevertheless, its role and underlying mechanism remain unclear in thyroid cancer. Here, we observed a significant upregulation of OIP5-AS1 in thyroid cancer tissues and cells, and upregulated OIP5-AS1 was correlated with poor prognosis in thyroid cancer. Moreover, OIP5-AS1 knockdown resulted in the inhibited cell proliferation and migration, while overexpressed OIP5-AS1 exhibited the reverse function in thyroid cancer. Besides, OIP5-AS1 was found to positively regulate Wnt/β-catenin signaling pathway. Through mechanism exploration, OIP5-AS1 was discovered to activate Wnt/β-catenin signaling pathway via FXR1/YY1/CTNNB1 axis. Finally, rescue assays indicated that the inhibitive role of silenced OIP5-AS1 in thyroid cancer cell growth and Wnt/β-catenin signaling pathway could be rescued by overexpression of CTNNB1 or addition of lithium chloride (LiCl). In conclusion, upregulation of OIP5-AS1 predicted unfavorable prognosis and enhanced thyroid cancer cell growth by activating Wnt/β-catenin signaling pathway.

## Introduction

As a type of endocrine malignancy, thyroid cancer contains a series of different histological types, such as primary thyroid sarcomas, papillary thyroid carcinomas, anaplastic thyroid carcinomas, primary thyroid lymphomas, follicular carcinomas, and medullary thyroid carcinomas.^1^^,^^2^ The morbidity of thyroid cancer keeps on growing rapidly worldwide.^3^^,^^4^ Previous studies showed that common therapeutic strategies, including radiation, chemotherapy, and surgery, are applied for thyroid cancer, but their treatment effects are not satisfactory.^5^, ^6^, ^7^ Additionally, the molecular mechanism regulating thyroid cancer remains poorly understood. Therefore, studies on molecular regulation mechanism and new therapeutic targets for thyroid cancer are in desperate need.

Long noncoding RNAs (lncRNAs) are identified as a class of endogenous cellular RNAs that have a length over 200 nucleotides and lack the ability to encode proteins.^8^^,^^9^ Increasing reports demonstrated that the abnormal expression of lncRNAs exhibits tumor-promotional or tumor-suppressive effect in various cancers.^10^^,^^11^ Importantly, lncRNAs modulate downstream gene expressions through the interaction of diverse biomolecules, such as DNA, RNA, and proteins.^12^ Moreover, recent evidence revealed that lncRNAs participated in regulating several cellular functions, containing cell cycle, proliferation, apoptosis, and differentiation.^13^^,^^14^ For example, lncRNA LINC00261 enhances cell apoptosis and hampers cell proliferation and invasion in choriocarcinoma.^15^ lncRNA AFAP1-AS1 facilitates thyroid cancer tumor growth and metastasis and restrains apoptosis.^16^ lncRNA OIP5-AS1 was found to play a carcinogenic role in a variety of cancers. As reported, OIP5-AS1 boosts cell proliferation and results in a poor prognosis in lung cancer.^17^ OIP5-AS1 sponges miRNA-129-5p and enhances the development of breast cancer via targeting SOX2.^18^ OIP5-AS1 exerts oncogenic function on biological behavior of glioma cells.^19^ Nonetheless, the functional role and molecular mechanism of OIP5-AS1 have not been researched in thyroid cancer.

Wnt/β-catenin signaling pathway was commonly reported to play a key role in the tumorigenesis and aggressiveness of human tumors, like colorectal cancer,^20^ glioblastoma,^21^ and pancreatic adenocarcinoma.^21^ Previous studies also demonstrated that existing lncRNAs are involved in the regulation of the Wnt/β-catenin signaling pathway in thyroid cancer,^22^^,^^23^ which suggests the pivotal role of Wnt/β-catenin signaling pathway in thyroid cancer. Although the association between some lncRNAs and Wnt/β-catenin signaling pathway has been revealed in thyroid cancer, the underlying regulation mechanism between OIP5-AS1 and Wnt/β-catenin signaling pathway is still needed to be further explored in thyroid cancer.

Here, we explored the function of OIP5-AS1 and the regulation mechanism between OIP5-AS1 and the Wnt/β-catenin signaling pathway. The results displayed that OIP5-AS1 activated Wnt/β-catenin signaling pathway via FXR1/YY1/CTNNB1 axis and then caused a poor prognosis and facilitated the proliferative and migratory of thyroid cancer cells. This discovery provided a meaningful revelation for exploring the potential therapeutic methods of thyroid cancer.

## Results

### Upregulation of OIP5-AS1 Could Predict Unfavorable Prognosis in Thyroid Cancer

To clearly explore the role of OIP5-AS1 in thyroid cancer, OIP5-AS1 expression in thyroid cancer tissues and cells (TPC-1, BCPAP, NIM, FTC-238, and FTC-133) was tested by conducting qRT-PCR. The normal matched tissues and normal thyroid follicular cells (Nthy-ori3-1) were taken as controls separately. As a result, OIP5-AS1 exhibited high expression in thyroid cancer tissues (Figure 1A). Similarly, OIP5-AS1 expression in thyroid cancer cell lines was also upregulated (Figure 1B). Among them, OIP5-AS1 level was highest in TPC-1 cell but was lowest in BCPAP cell. For this reason, we chose TPC-1 and BCPAP cells for the next experiments. Later, result from Kaplan-Meier analysis demonstrated that the sufferers with high OIP5-AS1 expression presented a more unfavorable survival time (Figure 1C). Next, we analyzed the correlation between OIP5-AS1 expression and clinical characteristics of thyroid cancer patients. OIP5-AS1 expression was revealed to be strongly associated with lymph node metastasis and clinical stages, but not with age or gender (Table 1). Based on the results of multivariate analysis, OIP5-AS1 expression and clinical stages were independent prognostic factors in thyroid cancer. Above results suggested the prognostic value of OIP5-AS1 in thyroid cancer (Table 2). Taken together, lncRNA OIP5-AS1 acted as a tumor facilitator in thyroid cancer.

**Figure 1:** OIP5-AS1 Predicted Poor Prognosis in Thyroid Cancer (A and B) OIP5-AS1 expression level in (A) tissues and (B) cell lines. (C) Kaplan-Meier analysis confirmed the association of OIP5-AS1 level with the prognosis of thyroid cancer patients. *p < 0.05, **p < 0.01.

**Table 1:** Clinical Characteristic and OIP5-AS1 Expression of Patients with Thyroid Cancer, (n = 60)

Variable	OIP5-AS1 Expression		p Value
	Low	High	
**Age**			

<45	16	13	0.606
≥45	14	17	

**Gender**			

Male	11	14	0.601
Female	19	16	

**Pathological Type**			

Papillary adenocarcinoma	10	12	0.789
Follicular adenocarcinoma	20	18	

**Lymph Node Metastasis**			

No	19	10	0.038*
Yes	11	20	

**Tumor Size**			

<3 cm	20	22	0.779
≥3 cm	10	8	

**Clinical Stages**			

I/II	17	8	0.035*
III/IV	13	22	

Low/high by the sample median. Pearson χ^2^ test. *p < 0.05 was considered statistically significant. The clinical data were evaluated by χ^2^ test.

**Table 2:** Prognostic Parameters in Thyroid Cancer Patients by Multivariate Analysis and Cox Regression Analysis

Variable	Category	p Value
Age		
	<45	0.311
	≥45	
Gender		
	Male	0.297
	Female	
Pathological type		
	Papillary Adenocarcinoma	0.285
	Follicular Adenocarcinoma	
Lymph node metastasis		
	No	0.787
	Yes	
Tumor size		
	<3 cm	0.683
	≥3 cm	
Clinical stages		
	I/II	0.007*
	III/IV	
OIP5-AS1 level		
	Low	0.034*
	High	

The prognostic value of OIP5-AS1 expression was showed by proportional hazards method analysis (p = 0.034). *p < 0.05 was considered statistically significant. Proportional hazards method analysis showed a positive, independent prognostic importance of OIP5-AS1 expression (p = 0.034). *p < 0.05, *p < 0.001 was considered statistically significant.

### OIP5-AS1 Enhanced Cell Growth in Thyroid Cancer

To validate this hypothesis, we knocked down OIP5-AS1 expression by transfecting sh-OIP5-AS1#1 and sh-OIP5-AS1#2, or upregulated OIP5-AS1 expression with the transfection of pcDNA3.1/OIP5-AS1 for the upcoming functional assays. As shown in Figures 2A and S1A, OIP5-AS1 expression was significantly silenced or overexpressed in both TPC-1 and BCPAP cells. Sh-OIP5-AS1#1 was selected for functional assays because of its higher transfection efficiency. Cell counting kit-8 (CCK-8) and 5-ethynyl-2′-deoxyuridine (EdU) immunofluorescence assays both manifested that OIP5-AS1 suppression inhibited, and OIP5-AS1 overexpression promoted the cell proliferation (Figures 2B and 2C; Figures S1B and S1C). Transwell assay elucidated that the migratory ability of TPC-1 and BCPAP cells was significantly inhibited by OIP5-AS1 knockdown and promoted by OIP5-AS1 overexpression (Figure 2D; Figure S1D). Above results indicated that OIP5-AS1 facilitated cell proliferative and migratory capacity in thyroid cancer.

**Figure 2:** OIP5-AS1 Enhanced Cell Growth in Thyroid Cancer (A) The transfection efficiency of sh-OIP5-AS1 and pcDNA3.1/OIP5-AS1 was assessed in TPC-1 and BCPAP cells. (B and C) CCK-8 assay and EdU assay were used to evaluate cell proliferation in response to OIP5-AS1 silence or overexpression (scale bar represents 100 μm). Histograms shown in (D) represent image quantification by ImageJ of three independent experiments for TPC-1 cell line. (D) Cell migration under OIP5-AS1 knockdown or overexpression was assessed by transwell assay. Histograms shown in (D) represent image quantification by ImageJ of three independent experiments for TPC-1 cell line. **p < 0.01, ***p < 0.001.

### OIP5-AS1 Activated Wnt/β-Catenin Signaling Pathway in Thyroid Cancer

In many studies, Wnt/β-catenin signaling pathway was proved to act critically in the modulation of cell proliferative ability and metastasis of cancers.^24^^,^^25^ For exploring whether OIP5-AS1 played an activated role in Wnt/β-catenin signaling pathway, experiments of luciferase reporter and western blot were carried out. In Figures 3A and S2A, TOP luciferase activity was considerably inhibited by OIP5-AS1 knockdown and promoted by OIP5-AS1 overexpression, whereas no significant change was showed in that of FOP group, indicating the activated function of OIP5-AS1 on Wnt/β-catenin signaling pathway in thyroid cancer. Later, this function was further elucidated by western blot and qRT-PCR assays. Genes of β-catenin, cyclin D1, and c-*myc* were correlated with Wnt/β-catenin signaling pathway. The results of qRT-PCR unveiled that their relative protein expressions were significantly downregulated in sh-OIP5-AS1 transfected cells and upregulated in cells transfected with pcDNA3.1/OIP5-AS1 (Figure 3B; Figure S2B). The same trend was also found after protein quantification in Figures 3C and S2C. Additionally, we discovered that the mRNA levels of CTNNB1, cyclin D1, and c-*myc* were reduced by OIP5-AS1 knockdown and increased by OIP5-AS1 overexpression (Figure 3D; Figure S2D). Immunofluorescence assay showed the knockdown of OIP5-AS1 inhibited the β-catenin nuclear translocation, while the reverse effect was observed in OIP5-AS1 overexpressed cells (Figure 3E; Figure S2E). The data strongly supported that OIP5-AS1 positively regulated Wnt/β-catenin signaling pathway.

**Figure 3:** OIP5-AS1 Activated Wnt/β-Catenin Signaling Pathway in Thyroid Cancer (A) TOP-FOP Flash assay was conducted to examine Wnt signaling activity upon OIP5-AS1 knockdown. (B) The protein levels of β-catenin, cyclin D1, and c-*myc* were detected after OIP5-AS1 knockdown. (C) The bands of western blot (WB)assays were quantified. (D) The function of OIP5-AS1 silence on the mRNA level of CTNNB1, cyclin D1, and c-*myc* was evaluated. (E) Immunofluorescence assay was performed to assess the role of OIP5-AS1 depletion in β-catenin nuclear translocation. *p < 0.05, **p < 0.01.

### OIP5-AS1 Interacted with FXR1

Next, the regulatory mechanism of OIP5-AS1 on Wnt/β-catenin signaling pathway was explored. Through the starBase website, fragile X mental retardation autosomal homolog 1 (FXR1) was predicted to be an RNA-binding protein for OIP5-AS1. FXR1 is a RNA-binding protein and upregulated in many cancers.^26^^,^^27^ To study the interaction between OIP5-AS1 and FXR1, we carried out RNA pull-down and RNA immunoprecipitation (RIP) assays. The results from RNA pull-down assay showed that FXR1 was notably enriched in the complex pulled down by OIP5-AS1 but not OIP5-AS1 antisense (Figure 4A). Furthermore, OIP5-AS1 expression was remarkably abundant in anti-FXR1 pellet in comparison to immunoglobulin G (IgG) control (Figure 4B). Through bioinformatics analysis, four potential binding sites between OIP5-AS1 and FXR1 were discovered. RIP results manifested that OIP5-AS1 combined with FXR1 in site 2 (Figure S3A). Further, the relative mRNA and protein expression levels of FXR1 were analyzed to be both decreased in sh-OIP5-AS1 transfected cells and increased upon OIP5-AS1 overexpression (Figures 4C and 4D). Additionally, a positive correlation between OIP5-AS1 and FXR1 expression was manifested in thyroid cancer tissues (Figure 4E). These data indicated that OIP5-AS1 bound to FXR1.

**Figure 4:** OIP5-AS1 Interacted with FXR1 and Could Regulate the Expression of FXR1 (A) Pull-down assay confirmed the interaction between OIP5-AS1 and FXR1 by using OIP5-AS1 sense biotin probe and OIP5-AS1 antisense biotin probe. (B) RIP assay showed the enrichment of OIP5-AS1 expression in anti-FXR1 precipitates. (C) The impact of OIP5-AS1 on FXR1 mRNA level was evaluated by qRT-PCR. (D) FXR1 protein level in sh-OIP5-AS1 transfected cells was evaluated by western blot. (E) Expression correlation between OIP5-AS1 and FXR1 in thyroid cancer tissues. **p < 0.01, ***p < 0.001.

### OIP5-AS1 Regulated YY1 Expression by Binding with FXR1

Through the starBase website, FXR1 was also predicted to be a RNA-binding protein for Yin Yang-1 (YY1). YY1 is a multifunctional transcription factor that could directly interacted with the promoter region of some genes and regulate their transcription.^28^^,^^29^ First, RNA pull-down and RIP assays were carried out to confirm the potential binding between YY1 and FXR1. It was proved that YY1 directly interacted with FXR1 (Figures 5A and 5B). For further analysis, the knockdown and overexpression efficiency of FXR1 were confirmed by qRT-PCR (Figure 5C). Subsequently, we observed that relative YY1 mRNA and protein levels were decreased in FXR1-silenced cells and increased upon FXR1 overexpression (Figures 5D and 5E). Besides, we found that FXR1 overexpression or knockdown abolished the effect of OIP5-AS1 on YY1 mRNA and protein levels (Figures 5F and 5G). Additionally, competition assay revealed that the interaction between OIP5-AS1 and FXR1 was inhibited by non-biotinylated OIP5-AS1 in a dose-dependent manner (Figure S3B). RIP assays further suggested that OIP5-AS1 knockdown inhibited the binding of FXR1 to YY1 (Figure S3C). Later, Pearson correlation analysis revealed the positive expression relationship between OIP5-AS1 and YY1 (Figure 5H). It was discovered that OIP5-AS1 expression was positively correlated with FXR1 or YY1 expression in thyroid cancer tissues from GEPIA database (Figures S3D and S3E). In general, OIP5-AS1 bound to FXR1 to regulate the expression of YY1.

**Figure 5:** OIP5-AS1 Regulated YY1 Expression by Binding with FXR1 (A and B) Pull-down and RIP analysis confirmed the interaction between YY1 and FXR1 by using YY1 sense biotin probe and YY1 antisense biotin probe. (C) Knockdown and overexpression efficiency of FXR1 were confirmed by qRT-PCR. (D and E) YY1 mRNA and protein levels were evaluated under FXR1 upregulation or downregulation. (F and G) YY1 mRNA and protein levels were detected in cells transfected the indicated plasmids. (H) The expression correlation between OIP5-AS1 and YY1 in thyroid cancer tissues was revealed. *p < 0.05, **p < 0.01, ***p < 0.001.

### YY1 Bound to the Promoter of β-Catenin

YY1 has been demonstrated to regulate gene expression at the transcriptional level and plays a notable part in biological processes of cancers.^30^^,^^31^ Through UCSC and JASPAR websites, YY1 was predicted to combine with CTNNB1 promoter. To confirm this, we performed chromatin immunoprecipitation (ChIP) assay, and results unveiled that the enrichment of CTNNB1 was obviously noticed in YY1 antibody (Figure 6A). Then, we separately knocked down or upregulated YY1 in thyroid cancer cell for the following experiments (Figure 6B). Through luciferase reporter assay, YY1 overexpression counteracted the suppressive effects of silenced OIP5-AS1 on the luciferase activity of CTNNB1 promoter (Figure 6C). According to qRT-PCR and western blot assays, both β-catenin mRNA (CTNNB1) and protein levels was reduced by transfecting sh-YY1 and increased in YY1 upregulated cells (Figures 6D and 6E). Additionally, the stability of CTNNB1 was weakened by YY1 depletion and enhanced by overexpression of YY1 (Figure 6F). It was further found that YY1 silence inhibited the β-catenin nuclear translocation whereas overexpressing YY1 promoted β-catenin nuclear translocation by performing immunofluorescence assay (Figure 6G). Conclusively, YY1 interacted with the promoter of CTNNB1 to regulate Wnt/β-catenin signaling pathway.

**Figure 6:** YY1 Bound to the Promoter of β-Catenin (A) ChIP assay certified the binding of YY1 to CTNNB1 promoter. (B) Transfection efficiency of pcDNA3.1-YY1 and sh-YY1 were determined by qRT-PCR. (B) Luciferase reporter assay was conducted to evaluate the luciferase activity of CTNNB1 promoter in cells transfected with indicated plasmids. (D and E) The effect of YY1 on β-catenin mRNA and protein levels were estimated. (F) The stability of CTNNB1 was measured after treating actD upon YY1 knockdown or overexpression. (G) The effect of YY1 on β-catenin translocation was determined by immunofluorescence (IF) assay. **p < 0.01.

### OIP5-AS1 Promoted Cell Growth of Thyroid Cancer via Wnt/β-Catenin Signaling Pathway

In order to verify whether OIP5-AS1 enhances the progression of thyroid cancer via Wnt/β-catenin signaling pathway, some restoration assays were designed and performed in TPC-1 cells. Lithium chloride (LiCl), an activator of Wnt/β-catenin signaling pathway was also employed for the follow-up experiments. As illustrated in Figure 7A, the reduced CTNNB1 expression in OIP5-AS1 downregulated cells was rescued by CTNNB1 upregulation. CCK-8 and EdU assays delineated that both pcDNA3.1/CTNNB1 transfection and LiCl treatment offset the suppressed cell proliferation in OIP5-AS1 downregulated cells (Figures 7B and 7C). What’s more, transwell assay implied that the inhibitive cell migration ability caused by OIP5-AS1 knockdown was restored through overexpressing CTNNB1 or adding LiCl (Figure 7D). We further discovered that β-catenin nuclear translocation decreased by OIP5-AS1 knockdown was rescued via transfecting pcDNA3.1/CTNNB1 or adding LiCl (Figure 7E). As shown in Figure 7F, the relative protein levels of Wnt/β-catenin signaling pathway were attenuated by OIP5-AS1 knockdown, whereas the inhibitive role could be rescued by overexpression of CTNNB1 or addition of LiCl. Therefore, OIP5-AS1 promoted cell growth of thyroid cancer via Wnt/β-catenin signaling pathway.

**Figure 7:** OIP5-AS1 Promoted Cell Growth of Thyroid Cancer via Wnt/β-Catenin Signaling Pathway (A) Results of qRT-PCR showed that OIP5-AS1 silencing-reduced CTNNB1 expression was rescued by overexpressing CTNNB1. (B and C) CCK-8 and EdU assay were performed to evaluate cell proliferation after transfecting the indicated plasmids (scale bar represents 100 μm). Histograms shown in (D) represent image quantification by ImageJ of three independent experiments for TPC-1 cell line. (D) The migration of cells transfected with shOIP5-AS1+pcDNA3.1, shOIP5-AS1+pcDNA3.1/CTNNB1, or shOIP5-AS1+LiCl was detected. Histograms shown in (D) represent image quantification by ImageJ of three independent experiments for TPC-1 cell line. (E) IF localization showed that OIP5-AS1 knockdown-inhibited nuclear translocation of β-catenin reversed by overexpression of CTNNB1 or addition of LiCl (scale bar represents 100 μm). (F) The protein levels of Wnt/β-catenin signaling pathway markers attenuated by OIP5-AS1 silencing were rescued by CTNNB1 overexpression or LiCl treatment. *p < 0.05, **p < 0.01.

### lncRNA OIP5-AS1 Boosted Tumor Growth *In Vivo*

To investigate whether OIP5-AS1 affected tumorigenesis *in vivo*, we subcutaneously injected nude mice with TPC-1 cells transfected with sh-NC, sh-OIP5-AS1, or sh-OIP5-AS1+pcDNA3.1/CTNNB1. After the experiment, the mice were euthanatized and then the tumors were dissected out. As shown in Figures 8A–8C, the size, volume, and weight of tumors in sh-OIP5-AS1 group were remarkably presented a lower level than that in sh-NC group, whereas the co-transfection of pcDNA3.1/CTNNB1 could rescue the repressive role of OIP5-AS1 knockdown. In addition, OIP5-AS1 level was significantly downregulated by OIP5-AS1 suppression in tumor tissues, whereas it could not be rescued by CTNNB1 overexpression. Furthermore, CTNNB1 expression in tumor tissues was significantly downregulated by OIP5-AS1 suppression, whereas the inhibition effect of sh-OIP5-AS1 could be partly counteracted by CTNNB1 overexpression (Figure 8D). Immunohistochemistry (IHC) assay showed that CTNNB1 overexpression significantly reserved OIP5-AS1 silencing-mediated suppression on OIP5-AS1 suppression (Figure 8E). Furthermore, positivity of Ki-67 and β-catenin was significantly decreased by OIP5-AS1 suppression, whereas the inhibition effect of sh-OIP5-AS1 could be partly counteracted by CTNNB1 overexpression (Figure 8F). Importantly, there was a positive correlation between OIP5-AS1 and β-catenin mRNA (Figure S3F). Above results suggested that OIP5-AS1 inhibition suppresses thyroid cancer tumorigenesis *in vivo*.

**Figure 8:** lncRNA OIP5-AS1 Boosted Tumor Growth *In Vivo* (A) The tumors were removed from the mice. (B and C) The growth curve and weight of tumors from mice were showed. (D) qRT-PCR analysis was used to evaluate the expressions of OIP5-AS1 and CTNNB1 in each group. (E) IHC was conducted to measure OIP5-AS1 expression in tissues collected from different groups of tumors (scale bar represents 50 μm). (F) IHC staining was used to test the positivity of Ki-67 and β-catenin in different groups (scale bar represents 50 μm). *p < 0.05, **p < 0.01.

## Discussion

Emerging studies have pointed out the versatile roles of lncRNAs in the biological process of numerous diseases, especially in cancers.^9^^,^^32^^,^^33^ lncRNA OIP5-AS1 was elucidated to exhibit oncogenic property in various cancers.^17^^,^^18^^,^^34^ In this work, significant upregulation of OIP5-AS1 was found in thyroid cancer tissues and cells. A previous study has reported that OIP5-AS1 could result in unsatisfactory prognosis in lung cancer.^17^ However, the specific function that OIP5-AS1 exerts on thyroid cancer hasn’t been explored so far. This research indicated that the upregulated OIP5-AS1 was correlated with poor prognosis in thyroid cancer. Additionally, suppression (or overexpression) of OIP5-AS1 resulted in a decrease (or increase) of cell proliferation and migration. All results uncovered that OIP5-AS1 presented oncogenic property in thyroid cancer.

Wnt/β-catenin signaling pathway is a typical signaling pathway that its abnormal activation was commonly studied on cancer initiation and progression. This pathway is in the involvement of regulating many cellular events, including cell differentiation, proliferation, and invasion through modulating the ability of β-catenin protein.^35^^,^^36^ As reported, Wnt/β-catenin signaling pathway exerts the regulatory role through the accumulation of β-catenin in the cytoplasm transferring to the nucleus and then its downstream genes were activated.^37^ The activated role of lncRNAs in Wnt/β-catenin signaling pathway has been reported in multiple cancers.^38^^,^^39^ Here, results showed that OIP5-AS1 promoted the nuclear translocation of β-catenin and positively regulated the signaling pathway, revealing that OIP5-AS1 boosted the progression of thyroid cancer through activating Wnt/β-catenin signaling pathway.

Subsequently, we focused on the regulatory mechanism of OIP5-AS1 operated on Wnt/β-catenin signaling pathway. FXR1, which was verified to combine with RNAs and thereby regulate their expression,^26^^,^^27^^,^^40^ was predicted to be a RNA-binding protein for OIP5-AS1. Mechanical experiments suggested that OIP5-AS1 could recruit FXR1. Meanwhile, FXR1 was also predicted to be a RNA-binding protein for YY1. We discovered that OIP5-AS1 bound with FXR1 to regulate YY1 expression. YY1 is a multifunctional transcription factor that can directly bind to a series of genes promoter region and regulate their transcription.^28^^,^^29^ For example, YY1 interacts with p65 to transcriptionally activate interleukin-6 (IL-6) and thereby increases IL-6 expression in microglial cells.^41^ YY1 promotes the expression of HDAC1 in hepatocellular carcinoma and reduces its sensitivity of to HDAC inhibitor.^42^ The binding site between YY1 and CTNNB1 was predicted by bioinformatics analysis. It was confirmed that YY1 bound to the promoter of CTNNB1 and positively regulate its expression, stabilization, and nuclear translocation. Rescue assays showed the inhibitive effect of OIP5-AS1 deficiency in thyroid cancer could be rescued by overexpression of CTNNB1 or addition of LiCl, which was consistent with the results *in vivo*. All the evidence supported OIP5-AS1 activated Wnt/β-catenin signaling pathway through FXR1/YY1/CTNNB1 axis.

This work was the first to reveal the role and regulatory mechanism of OIP5-AS1 in thyroid cancer. Additionally, other regulatory mechanisms of OIP5-AS1 in thyroid cancer should be explored in the future. The above results revealed that OIP5-AS1 acted as an oncogenic lncRNA that activated Wnt/β-catenin signaling pathway through FXR1/YY1/CTNNB1 axis in thyroid cancer. Hence, OIP5-AS1 may bring new insights into the exploration of thyroid cancer treatment.

## Materials and Methods

### Clinical Samples

60 pairs of thyroid cancer tissues and paired normal tissues were all provided by Sun Yat-sen University Cancer Center. Tissues were all kept in liquid nitrogen before the experiments. The patients who provided above tissues had never received any tumor-specific treatment. The Ethics Committee of Sun Yat-sen University Cancer Center approved this study, and written consent was signed by all patients.

### Cell Culture

Human thyroid cancer cell lines (TPC-1, BCPAP, NIM, FTC-238, FTC-133), along with normal thyroid follicular cell line (Nthy-ori3-1) were used in our study. The above cell lines were procured from American Type Culture Collection (ATCC, Manassas, VA, USA). Dulbecco’s modified Eagle’s medium (DMEM; Invitrogen-GIBCO, Carlsbad, CA, USA) was used to culture TPC-1, BCPAP, FTC-238, and FTC-133 cells, while RPMI 1640 (Invitrogen-GIBCO) was applied to culture NIM and Nthy-ori 3-1 cells. Both mediums were supplemented with 10% FBS, 1% penicillin/streptomycin, and contained 5% CO_2_ at 37°C. Actinomycin D (actD), a polypeptide antibiotic, binds to DNA to inhibit RNA and protein synthesis. For actD treatment, 1 × 10^5^ cells were placed in 96-well plates for incubating 24 h. Later, 6 mL complete medium containing 10 μg/mL actD was added, and DMSO was taken as a control. LiCl, a classical Wnt pathway activator, was also applied to treat thyroid cancer cells at the concentration of 20 mM.

### Cell Transfection

For knockdown of OIP5-AS1, FXR1, or YY1, short hairpin RNAs (shRNAs) targeted to OIP5-AS1, FXR1, or YY1 were transfected into thyroid cancer cells. Non-targeted shRNA was used as negative control (sh-NC). To overexpress OIP5-AS1, FXR1, YY1, or CTNNB1, we separately cloned an entire sequence of these genes into pcDNA3.1 vector (named as pcDNA3.1/OIP5-AS1, pcDNA3.1/FXR1, pcDNA3.1/YY1, or pcDNA3.1/CTNNB1). Empty vector was taken as a negative control (pcDNA3.1). According to the proposals of the manufacturer, Lipofectamine 2000 Reagents (Invitrogen, Carlsbad, CA, USA) were applied to transfect these plasmids into TPC-1 and BCPAP cells. For transfection in 6-well plates, 2 μg plasmids, and 6 μL transfection reagent (Lipofectamine 2000) were placed into per well, and then incubated for 6 h with 5% CO_2_ at 37°C.

### qRT-PCR

TRIzol (Invitrogen, Carlsbad, CA, USA) was employed to extract the RNAs from cells. Reverse Transcript Kit (Applied Biosystems, Foster City, CA, USA) and Taqman Advanced miRNA cDNA Synthesis Kit (Waltham, MA, USA) were used to implement reverse transcription. SYBR Green Master Mix kit (Takara) was applied for qRT-PCR assay. GAPDH was considered as the internal reference. At last, the data were analyzed with the use of 2^−ΔΔCt^ method. The primer sequences were as listed:

OIP5-AS1: 5′-TGCGAAGATGGCGGAGTAAG-3′ (forward) and 5′-TAGTTCCTCTCCTCTGGCCG-3′ (reverse);
FXR1: 5′-CCCTAATTACACCTCCGGTTATG-3′ (forward) and 5′-TCTCCTGCCAATGACCAATC-3′ (reverse);
YY1: 5′-AGAATAAGAAGTGGGAGCAGAAGC-3′ (forward) and 5′-ACGAGGTGAGTTCTCTCCAAT-3′ (reverse);
CTNNB1: 5′-TGCAGTTCG-CCTTCACTATG-3′ (forward) and 5′-ACTAGTCGTGGAATG-GCACC-3′ (reverse);
GAPDH: 5′-GAAGGTGAAGGTCGGAGTC-3′ (forward) and 5′-GAAGATGGTGATGGGATTTC-3′ (reverse).

### CCK-8 Assay

1 × 10^3^ cells of TPC-1 and BCPAP were incubated in 96-well plates for 1, 2, 3, or 4 days at 37°C after being transfected. Afterward, 10 μL of CCK-8 solvent was supplemented to every well for extra 4 h of incubation. A microplate reader was utilized to observe the absorbance at 450 nm.

### Bioinformatics Analysis

Through starBase website (http://starbase.sysu.edu.cn/), FXR1 was predicted to be an RNA-binding protein for OIP5-AS1 YY1. YY1 was predicted to be a potential upstream transcription regulator for CTNNB1 by using online database UCSC (http://genome.ucsc.edu/) and JASPAR (http://jaspar.genereg.net/).

### RIP Assay

Cells were isolated and lysed with RIP buffer supplemented with RNase inhibitor. 100 μL extracted cells was cultured in RIP buffer, which contains anti-FXR1 coated on magnetic beads. The precipitated RNAs were eluted and then tested by utilizing qRT-PCR. Input and IgG served as controls.

### RNA Pull-Down Assay

To detect the binding ability, OIP5-AS1, OIP5-AS1 antisense, YY1, and YY1 antisense were biotinylated by Biotin RNA labeling mix (Roche Diagnostics, Indianapolis, IN, USA). Biotinylated RNA was co-incubated with cell lysate containing streptavidin beads. After incubation of 1 h, proteins were eluted and detected with the application of western blot.

### Luciferase Reporter Assay

For TOP/FOP Flash assay, cells of TPC-1 and BCPAP were planted in 24-well plates and with the co-transfection of TOP/FOP Flash reporter vectors (Biovector). A number of copies of TCF/LEF DNA binding sites were cloned into firefly luciferase reporter system vectors to construct TOP-Flash vectors. Control plasmids contained mutant TCF/LEF DNA binding sites, namely FOP-Flash vectors. The promoter region of CTNNB1 was cloned with pGL3 luciferase reporter vector (Promega Corporation, Madison, WI, USA). TPC-1 and BCPAP cells in 96-well plates were co-transfected with above vector and sh-OIP5-AS1, sh-OIP5-AS1+pcDNA3.1/YY1, or sh-NC for 48 h. Afterward, the luciferase activities were tested via luciferase assay kit (Promega, Madison, WI, USA).

### Immunofluorescence

The transfected cells were plated into 6-well plates. The cells were fixed through the employment of 4% paraformaldehyde, infiltrated with the application of 0.2% Triton X-100, cultured through the employment of 3% hydrogen peroxide solution under the environment without light, and sealed with the application of 5% bovine serum albumin (BSA), followed by being incubated with primary antibodies solutions at 4°C overnight. The primary antibodies were anti-β-catenin (ab16051). Next day, after removing the primary antibodies solutions, the transfected cells were cultured with secondary antibody solution, followed by being stained with DAPI. The images were photographed employing a fluorescence microscope.

### Western Blot

Radioimmunoprecipitation assay (RIPA) lysis buffer (Beyotime Biotechnology, China) was applied to lysed cells. Then, total extracted protein was isolated by 10% SDS-PAGE and immediately transferred onto polyvinylidene fluoride (PVDF) membranes (GE Healthcare Bio-Sciences, Piscataway, NJ, USA). Afterward, the membranes were incubated using primary antibodies of FXR1 (ab129089), CTNNB1 (ab16051), cyclin D1 (ab16663), c-*myc* (ab32072), and GAPDH (ab8245). All primary antibodies were purchased from Abcam Company (Abcam, Cambridge, UK). Then the membranes were appropriately incubated using secondary antibodies. Finally, blots were imaged by ECL detection reagents (Amersham Biosciences, Sweden).

### Transwell Assay

Transfected cells were placed in the upper transwell chamber. Afterward, 600 μL of DMEM medium containing 10% FBS (Hyclone, Shanghai, China) was supplemented into the lower chamber. 24 h later, cells were fixed and stained separately using methanol and crystal violet on the lower chamber. The quantity of migrated cells was calculated through inverted microscope (IX71, Olympus, Tokyo, Japan).

### EdU assay

In EdU assay, cells of TPC-1 and BCPAP were incubated with EdU solution for 2 h, and then immobilized by PBS, which contains 4% paraformaldehyde. Subsequently the cells were transferred into 70% ethanol and then stained. Eventually, cells were visualized by fluorescence microscopy.

### ChIP Assay

ChIP assay was conducted with the application of EZ-CHIP KIT (Millipore, Billerica, MA, USA). Formaldehyde was added to treat the cells to build DNA-protein cross-links. Afterward, chromatin fragments were generated after the sonication of cell lysates. Anti-YY1 and anti-IgG were used for immunoprecipitating chromatin fragments. Lastly, the precipitated chromatin DNA was analyzed by qRT-PCR.

### *In Vivo* Experiment

Male BALB/c nude mice aged 5–6 weeks were provided by the Shanghai LAC Laboratory Animal (Shanghai, China). To evaluate the tumorigenic effects *in vivo*, we subcutaneously injected cells (1 × 10^6^ cells per mouse) with the transfection of sh-NC, sh-OIP5-AS1, and sh-OIP5-AS1+pcDNA3.1/CTNNB1 into the flanks of the mouse (n = 5 per group). After a month, the mice were euthanized. Then the tumors were acquired and weighed. The volume of tumors was calculated as length × (width^2^/2). All procedures in the experiment were carried out with the approval of Sun Yat-sen University Cancer Center.

### IHC and *In Situ* Hybridization (ISH)

IHC staining of Ki-67 and β-catenin was carried out in accordance with previous study.^43^ Incubated with goat anti-rabbit secondary antibody (Vector Laboratories, CA, USA), slides were incubated with Ki-67 and β-catenin antibodies (Cell Signaling Technology) overnight at 4°C. For visualization, Tris-HCl buffer containing 3, 30-diaminobenzidine, and 0.1% H_2_O_2_ was applied to incubate slides. Finally, Hematoxylin QS (Vector Laboratories) was used for counterstaining.

Expression of OIP5-AS1 in thyroid cancer was assessed by using biotin-labeled OIP5-AS1 ISH probes (BOSTER, Wuhan, China). Briefly, after the immobilization with 4% paraformaldehyde and incubation with Proteinase-K, the slides were hybridized with 200 nM of OIP5-AS1 probe for 40 min at 50°C. Then, diaminobenzidine (DAB) solution (BOSTER) was used for visualization of probe signal.

### Statistical Analysis

Statistical analysis was conducted with the employment of SPSS 17.0 statistics software (SPSS, Chicago, IL, USA). Data were shown as the mean ± standard deviation (SD). Each experiment was conducted more than 3 times. Overall survival curves were analyzed through Kaplan-Meier method and the log-rank test. Pearson correlation analysis was utilized to detect the expression correlations. The differences between groups were calculated by Student’s t test or one-way ANOVA test. p < 0.05 was regarded with statistical significance.

## Conflicts of Interest

The authors declare no competing interests.

## Supplemental Information

Document S1. Figures S1–S3 and Supplemental Files

Document S2. Article plus Supplemental Information
